# Biomechanical Research on Special Ability of Long Jump Take-Off Muscle Based on Multisource Information Fusion

This article has been retracted.

**DOI:** 10.1155/2022/2556087

**Published:** 2022-04-07

**Authors:** Yue Ren, Bingquan Luo, Jun Chu

**Affiliations:** Capital University of Physical Education and Sports, Beijing 100191, China

## Abstract

For athletes of different sports, their muscle activities in different sports will show different special characteristics according to different sports. The purpose of this paper is to study the technology of multi-information fusion and to study the athletes of the long jump competition. The relevant research on the muscle specific ability test methods of the athletes in the long jump competition is of great significance to the study of the long jump. This paper proposes a long jumper's special muscle ability experiment, using the now very popular multi-information fusion technology, to conduct in-depth research on the biomechanics of the long jumper's special ability of the take-off muscle, which can provide an effective scientific basis for the special ability level and special strength of the long jumper's take-off sports. The results of the study show that the hip joint of the take-off leg produces greater hip extensor torque during the take-off action of long jump, and the active contraction ability of the knee flexor group is very important for taking off and avoiding damage to the posterior femoral muscle group. The change range of the pressure center is between 51.26% and 74.35%, which has great application value in actual training.

## 1. Introduction

Multi-information sensing technology is one of the most popular research technologies nowadays. Since the technology came out in the late 1950s, in the past 60 years, due to its advantages in accuracy, consistency, and fault tolerance, countries around the world have eyes turned to this technology. This technology has been applied in military and civilian fields, and the multisensor fusion sensing technology to solve the problem that a single sensor is prone to failure has become a research hotspot. Long jump is composed of four parts: running, taking off, flying, and landing, and taking off is one of the main links and important contents of long jump technology research. The long jump and sprint are performed by athletes who maintain high speed. The characteristics of the long jump competition determine the contraction method and characteristics of the joint muscles of the lower limbs during the long jump. The different abilities of each muscle group are embodied, which can represent the unique ability of athletes to a certain extent. Therefore, in the process of taking off, it is undoubtedly very important for the rapid strength and the ability to exercise the rising and swinging leg joint muscle groups.

My country's multi-information fusion technology is mainly used in robot development, and the multi-information fusion technology used in long jump is still in the theoretical stage. Multi-information fusion systems are basically divided into three types, namely, mathematical models, functional models, and structural models. Among them, the mathematical model uses different mathematical methods to process the data to complete the data merging, while the functional model is generated from the basic data fusion unit and the fusion system in the module, and the structural model deals with the interaction between different structures. Based on the current biomechanical analysis of long jump technology, although some studies have analyzed the activity of each joint muscle group, they mainly focus on the movement mode of each link, without qualitative analysis of the anatomical function of the muscles and joints. And in analyzing the dynamics of each joint, there are few studies on science and the role of individual joint muscle groups in exercise technology. But research in this area is very important for specific exercise techniques and specific strength training and has very important research value and significance.

Multi-information fusion technology is one of the most popular information fusion technologies. It is widely used in education, sports, finance, and other industries and has very important research value and significance. Long jump is a very ancient sport. It has evolved gradually from ancient people chasing prey, and it occupies a very important position in modern sports. Among them, the research on long jump has been hotly discussed by scholars at home and abroad. In order to test the actual situation in the long jump, Yoshida et al. quantitatively evaluate the long jump using two analysis items. In the long jump, the take-off index is defined as the vertical speed value during the take-off divided by the deceleration of the horizontal speed in the take-off movement. The teaching of the rhythm of the last three steps of the approach run is invalid for the long jump [1]. For athletes with under-knee amputations (BKA), the biomechanical knowledge of long jump take-off steps is not comprehensive, but it is important for improving training programs and performance. Funken found that compared with other BKA athletes, those BKA athletes who performed better in the long jump had relatively higher changes in the individual internal joint angles of the knee and hip joints at the moment of take-off compared with nonamputation athletes [2]. In order to reveal the effect of segmental rotation on the vertical speed and the horizontal speed loss during the take-off of the long jump, Sado et al. use a 3D motion capture system and a force plate to capture the athlete's long jump. Although calf and thigh movements involve a loss of horizontal speed, the elevation of the free leg side of the pelvis produces vertical speed without loss of horizontal speed. This research provides evidence for a new long jump technique method [3]. In order to conduct research on excellent long jump events, Gaspar et al. analyzed the mechanical properties (muscle strength and tendon stiffness) of the triceps (TS) tendon unit (MTU) of outstanding jump athletes (long jump, triple jump, high jump, and pole vault) and monitored the changes in these characteristics caused by training jumpers within one year to detect the potential changes in the uniformity of adaptation within the TS MTU [4]. Reinforced long jump training with progressive load can improve motivation and sports swimming start parameters. Rebutini et al. aim to determine the impact of the enhanced long jump training program on the torque around the joints of the lower limbs and the dynamics and kinematics parameters during the beginning of the swimming jump. The enhanced long jump training program can effectively enhance the torque around the joints of the lower limbs and control the direction of the composite vector. Coaches should use long jump training instead of vertical jump training to improve swimming starting performance [5]. Compared with the leg focus, the arm focus leads to a significantly larger jump distance, but there is no difference in the projection angle. Coker extended these findings to teenagers and revealed differences in projection angles, indicating that prompting teenagers to focus on arm movements does not seem to restrict movement in the same way as adults [6]. In order to determine the biomechanical factors that limit the distance and the best effort stand-up long jump technique, Yokozawa et al. determined the limiting factors and jumping technique by analyzing the relationship between the joint strength mode of the propulsion stage of the standing long jump and the maximum isokinetic strength of the lower limbs. This phenomenon may originate from the strategy of enhancing the strength of the lower limbs through the coupling of reverse movement and arm swing with the movement of the lower limbs [7]. Although the above-mentioned related studies are conducted by well-known research scholars at home and abroad, they have not used new techniques to conduct detailed research on the ancient movement of long jump. There is sufficient theoretical support in theory, and a large number of them have also been carried out.

Long jump is a very old sport that evolved in the process of primitive humans catching prey. It has been loved by people for thousands of years, but it has not been studied and applied in practice until modern times. This article uses multisource information fusion technology to study the long jump and uses multiple experiments and data to observe the muscle changes during the take-off of the athletes in the long jump. The actual experimental results are recorded, which is different from the previous researchers at home and abroad. Yes, this experiment uses the more popular multi-information fusion technology for research. Based on the biological basis of previous related research, using the current relevant experimental data, the biological characteristics of the muscle specific ability of different telemobilization during the long jump are carried out. Research has great practical application and research value in actual sports events.

## 2. Multisource Information Fusion Technology to Study the Biological Changes of Long Jump Take-Off Muscles

### 2.1. Multisource Information Fusion Technology

Multisource information fusion technology is the so-called multisensor information fusion (MSIF), which is the process of using computer technology to process information and data from multiple sensors or multiple sources. Multisensor information fusion is used to information processing technology of multiple or multiple sensors in different locations [8]. Multisource information fusion technology is to sort out information from multiple sources and summarize it to a certain place. Through multisource information fusion technology, information integration can be promoted. With the development and maturity of sensor application technology, data processing technology, computer software and hardware technology, and industrial control technology, multisensor information fusion technology has become a popular emerging subject and technology. And it is believed that with the advancement of science, multisensor information fusion technology will become a specialized technology for comprehensive processing and research of intelligent and refined data, information, and images [9]. The basic principle of multisensor information fusion technology is like the process of the human brain's comprehensive information processing. Various sensors are processed for multilevel and multispace information complementation and optimized combination processing, and finally, a consistent interpretation of the observation environment is produced. In this process, it is necessary to make full use of multisource data for reasonable control and use, and the ultimate goal of information fusion is to derive more useful information through the multilevel and multifaceted combination of information based on the separated observation information obtained by each sensor [10]. This not only takes advantage of the cooperative operation of multiple sensors but also comprehensively processes data from other information sources to improve the intelligence of the entire sensor system, as shown in Figure 1.

The greatness of the sensor integration concept is that it receives input from different sensors and sensor types, can perform different processing according to different input data, and use the combined information to understand the environment more accurately [11]. Compared with a standalone system, the system can make better and safer decisions. The data fusion technology originated from the sonar signal processing system funded by the US Department of Defense in 1973. With the extensive development of information technology in the 1990s, a broader concept of “data” was proposed [12]. MSDF Multisensor Data Fusion technology emerged at the historic moment. The main advantage of data integration is to make full use of multisensor data sources at different times and locations, analyze, integrate, control, and operate in accordance with certain standards. [13]. Obtain a consistent interpretation and description of the measured object, and then realize the corresponding decision-making and estimation, so that the system can obtain more sufficient information than its various components [14]. The first is the establishment of a multisource sensing system and calibration, then collect data and perform digital signal conversion, then perform data preprocessing and feature extraction, followed by calculation and analysis of the fusion algorithm, and finally output stable, more sufficient and consistent target feature information, multisource information fusion. The detailed schematic diagram of the technology is shown in Figure 2.

In the multi-information fusion technology, Chinese medicine uses multiple sensors to collect corresponding various external information. For the convenience of related research, it is necessary to use multiple cameras to collect different information. For the commonly used pinhole camera model, the relationship between the three-dimensional world point *M* and its projection point *m* on the image is [15]

(1) $$\begin{array}{c} \text{s}\tilde{\text{m}}=A\left[\text{Rt}\right]\tilde{M}. \end{array}$$

In the formula, *s* represents the size scaling factor, and the transformation matrix [Rt] is the external parameter of the camera. The rotation and translation are realized by the matrices *R* and *t* [16]. *A* is the internal parameter matrix, specifically,

(2) $$\begin{array}{c} A=\left[\begin{array}{ccc} \alpha & \gamma & u_{0}\\ 0 & \beta & v_{0}\\ 0 & 0 & 1 \end{array}\right]. \end{array}$$

Without loss of generality, for the convenience of research, assuming that the *Z* axis is always 0, then expand the formula (1) to obtain

(3) $$\begin{array}{c} s\left[\begin{array}{c} u\\ v\\ 1 \end{array}\right]=A\left[r_{1}\;r_{2}\;r_{3}\right]\left[\begin{array}{c} X_{W}\\ Y_{W}\\ Z_{W} \end{array}\right]=A\left[\begin{array}{ccc} r_{1} & r_{2} & t \end{array}\right]\left[\begin{array}{c} X_{W}\\ Y_{W}\\ 1 \end{array}\right]. \end{array}$$

Therefore, the pinhole model can be further expressed as follows:

(4) $$\begin{array}{c} \left\{\begin{array}{c} \text{s}\tilde{\text{m}}=\text{H}\tilde{\text{M}}\\ H=A\left[\begin{array}{ccc} r_{1} & r_{2} & r_{3} \end{array}\right] \end{array}\right. \end{array}$$

Suppose there is a value whose mean is 0 and the covariance matrix is *C*_*i*_. Through the following objective function we can get the maximum likelihood estimate of the *H* matrix:

(5) $$\begin{array}{c} \underset{i}{\sum }\left(m_{i}-\hat{m_{i}}\right)C_{i}^{-1}\left(m_{i}-\hat{m_{i}}\right). \end{array}$$

The relevant parameters in this formula are defined as

(6) $$\begin{array}{c} \hat{m_{i}}=\frac{1}{\bar{h_{3}^{T}\hat{m_{i}}}}\left[\begin{array}{c} h_{3}^{T}M_{i}\\ h_{3}^{T}M_{i} \end{array}\right]. \end{array}$$

Because the image processing process of each information source does not interfere with each other in practice, it is usually assumed to be

(7) $$\begin{array}{c} C_{i}=\delta^{2}I. \end{array}$$

Therefore, the problem of camera calibration can be transformed into a nonlinear problem of quadratic programming:

(8) $$\begin{array}{c} \min\underset{i}{\sum }\left|\left|m_{i}-\hat{m_{i}}\right|\right|. \end{array}$$

In the actual shooting, the corresponding relationship between the camera pitch angle *θ* and the actual height of the image center mapped to the calibration board and the difference between the two movement distances of the calibration board is as follows:

(9) $$\begin{array}{c} \theta =\arctan\frac{h_{1}-h_{2}}{s_{2}} \end{array}$$

The actual installation position of the camera in the multisource information sensing technology can be obtained through a simple trigonometric function relation:

(10) $$\begin{array}{c} \left\{\begin{array}{c} \tan\theta =\frac{H-h_{1}}{S}\\ \tan\left(\alpha -\theta \right)=\frac{H-h}{S} \end{array}\right.. \end{array}$$

Simplify the above formula to get

(11) $$\begin{array}{c} \left\{\begin{array}{c} H=h+\frac{\left(h-h_{1}\right)\left(\tan\theta -\tan\alpha \right)}{\tan\left(1+\sin^{2}\theta \right)}\\ S=\frac{H-h}{\tan\theta -\text{s}} \end{array}\right.. \end{array}$$

Multi-source information fusion is based on multiple (same or heterogeneous) information sources. From the fusion level, the fusion model usually performs information fusion processing from three levels of data, features, and decision-making [17]. The system structure using information fusion technology can generally be divided into centralized fusion, distributed fusion, and hybrid fusion architecture. For practical problems, according to the differences in the characteristics of the information source data, different levels of fusion methods can be used alone or a combination of two levels of progressive fusion methods can be used to obtain a fusion scheme with better system performance [18, 19]. The basic principle and starting point of the concept of information fusion is as follows: make full use of multiple information sources, and combine the redundant or complementary information of multiple information sources in space or time according to specific standards to obtain a consistent interpretation of the measured object or describe, make the information system have better performance compared to the system composed of the various subsets contained in it, where the data refers to the measurement data collected by the sensors of each section. The tissue structure and biological properties of muscle determine its function, and the change of muscle function also affects its structure. The specific key technology of multisource information fusion is shown in Figure 3.

### 2.2. Long Jump Take-Off Method

Long jump (long jump), which can also be called “rapid long jump”, is a very old track and field sport. Athletes run in a straight line from a run-up to a straight line. During the running in, one foot jumps in the air, and finally, both feet fall. A sport of entering a bunker, in the end, the referee decides whether to win or lose through the distance in the bunker [20]. Long jump was originally a life skill for primitive humans to hunt for food and escape from wild animals and later became a condition and method for recruiting, selecting, and training soldiers. First of all, the selection of the long jump athlete needs the athlete's physical quality, strong and powerful thigh muscles and arm muscles, by looking at the performance of the athletes through the trial jump. In the ancient Greek Olympics, the long jump has become one of the official events and has always been welcomed and loved by people [21]. The modern long jump originated in the United Kingdom. The 1896 Athens Olympics confirmed the men's long jump as an official event. In 1935, American athlete, Jesse Owens broke the 8-meter mark with a height of 8.13 meters. In 1948, the women's long jump was included in the official event of the London Olympics. The world's highest organization for long jump is the World Athletics Association, which was established in 1912 and has a long history of more than one hundred years [22]. The main responsibility of this federation is to develop the world's track and field sports, specify the timing method of track and field competitions, and record new world records for track and field events. The long jump consists of four parts: approach, take-off, flight, and landing. Among them, the take-off action is one of the main links and important contents of technical research in long jump sports. The take-off action in the long jump is the athlete making longer jumps while maintaining high-speed movement, while the horizontal speed of the human body during the take-off of elite athletes (jump length 8 ~ 8.95 m) reaches 9 ~ 11.2 mös, and the horizontal speed of the center of gravity at the end of the take-off action is also 8 ~ 10mös, the athlete's take-off time is 0.1 ~ 0.14 s [23]. The characteristics of the long jump competition determine the way of long jump contraction and the characteristics of the joint muscles of the lower limbs. In the approach stage of the long jump, push your feet on the ground quickly and forcefully. At the same time, bend your arms slightly, swing from back to front and up, jump up and take off, and fully spread your body. Athletes are required to complete the speed increase at a high speed. Each muscle group in the joints quickly shows signs of various contractions, reflecting the different capabilities of each of these joint muscle groups. During the take-off action, rapid swing, muscle strength, and physical ability are the performances that affect the joint muscle groups of the take-off leg. The coordination and cooperation of various body organizations in the entire long jump is undoubtedly very important, as shown in Figure 4. Shown are the four components of long jump.

### 2.3. Muscle Specific Ability Biomechanics

Muscles are muscles (skeletal muscles) which are an important part of the human movement system and the power source of human movement. It can be said that muscle is also the most attractive research field in biomechanics research [24]. The strength factor is especially the burst force capacity of the muscle group of the lower limbs and puts forward a higher requirement on the strength of the ankle joint. Because the last point of force in the standing long jump is the forefoot (or even the toe), the plantar-flexion force of the ankle joint is required to have a considerable strength. The mechanical properties of muscles are very complicated. It is related to the mechanical properties of various components of muscles. So far, it is still under continuous research and exploration. Muscle tissue structure and biological characteristics determine muscle function, and changes in muscle function will also affect its structure. Therefore, studying muscle tissue structure and biology is one of the foundations for studying muscle biomechanical characteristics. In order to reflect the biomechanical characteristics of muscles, the establishment of a model is used to describe muscle mechanical characteristics. Muscle tissue structure and biological characteristics determine muscle function, and changes in muscle function will also affect its structure [25]. Therefore, studying the structure and biology of muscle tissue is one of the foundations for studying the biomechanical characteristics of muscles. In order to reflect the biomechanical characteristics of muscles, the establishment of a model is used to describe the mechanical characteristics of muscles. The anterior calf muscle group, in the landing buffer stage for centripetal contraction and in the pedal extension stage for centrifugal contraction, its role is dorsiflexion of the ankle joint, which participates in the take-off leg in the landing buffer process of pressing down the landing buffer action and with the back side muscle group of the pedal extension action. The schematic diagram of the human skeletal muscle model is shown in Figure 5.

According to the dynamics of the human body and various joints, it is used to calculate the dynamics of each lower extremity joint during the human body movement, and the relevant knowledge of inverse dynamics is used for detailed explanation. The movement direction of the body link of the ground movement is upward, that is, hip joint, knee joint, from flexion to extension, ankle from dorsiflexion to plantar flexion, the direction of gravity is downward, the muscle group involved in the movement completes the centripetal work, and the direction of muscle force is consistent with the direction of trunk movement. The specific content includes the plantar during the take-off process, the reaction force and relative volume of the support, the duration of the muscles in the take-off process, and the relative volume of the hip, knee, and ankle joints [26]. According to Newton's second law:

(12) $$\begin{array}{c} m\frac{d^{2}y}{dt^{2}}=\sum Ey,\\ m_{1}\ddot{y}c_{1}+m_{2}\ddot{y}c_{2}=\text{GRFy}+\text{Fe}-\left(m_{1}+m_{2}\right)g, \end{array}$$

(13) $$\begin{array}{c} \text{GRFy}=m_{1}\ddot{y}c_{1}+m_{2}\ddot{y}c_{2}+\left(m_{1}+m_{2}\right)g-\text{Fe}. \end{array}$$

The impulse can be calculated by integrating the GRFy in the time of the take-off action of the long jump. The specific formula is

(14) $$\begin{array}{c} Iy=\int_{t1}^{t2}\text{GRFy}∙\text{dt}. \end{array}$$

In the actual experiment, the treadmill is used, and the specific friction coefficient between the track and the running belt is known, so that the friction between the running belt and the running platform during the stepping process is

(15) $$\begin{array}{c} \text{fu}=\text{GRFy}∙\mu . \end{array}$$

The formula for calculating the friction coefficient is, assuming that the friction coefficient does not change with the speed of the running belt,

(16) $$\begin{array}{c} \mu =\frac{\text{fm}}{N}. \end{array}$$

In combination with Newton's second law, we can get

(17) $$\begin{array}{c} {\text{m}}_{\text{e}}\text{a}=\text{fk}-\text{GRFx}-\text{fu}-\text{fs}. \end{array}$$

After simplification, GRFx can be calculated, the formula is as follows:

(18) $$\begin{array}{c} GRFx=fk-m_{e}a-fu-fs. \end{array}$$

Finally, the calculation is based on the fixed rotation force. When the foot falls on the treadmill, the horizontal force received by the foot is provided by the running belt. The main part of the horizontal force is the inertial force of the rotating system.

(19) $$\begin{array}{c} \sum M=I∙\beta . \end{array}$$

## 3. Experiment on Biological Changes of Take-Off Muscles in Long Jump

### 3.1. Development of an Experimental Test System for the Special Ability of the Jumping Leg

In competitive sports, physical fitness is an important part of whether an athlete is competitive, and different competitive sports have different attributes. The exercises used in actual exercises to develop motor skills and basic motor skills required for the competition are called special exercises. If this type of exercise is close enough to the actions of a formal competition, it may play a role in training athletes. From a biomechanical point of view, these exercises must follow the principle of dynamic adaptation, that is, compatible with competitive competitions in the following five aspects: range and direction of motion, significant effective range and direction of motion, force (or muscle strength), maximum movement speed, muscle function status. Regardless of the five aspects, specific exercises can be fully adapted to the competitive functions of the above five areas. The choice of specific training courses should be as basic as possible but adapt to the intensity of the competition. The long jump consists of four consecutive stages: approach, take-off, flight, and landing. In the whole long jump, the take-off is the most important link. Because it is this stage that produces the vertical speed that causes the body to leave the ground, which can lift the body for a period of time. When starting a long jump, the athlete must make full use of the speed gained from the approach to create the highest possible starting speed and take-off angle in the shortest possible time. The specific technique of the take-off action is divided into three stages: take-off foot landing, cushioning, and stretching. According to the particularity of the special ability training of long jump, it is used to develop and improve the special ability of long jump lower limbs, including the ability of eccentric contraction and concentric contraction, which can give full play to the energy of the athlete's body.

In this experiment, we selected 8 outstanding male long jumpers from the physical education department of the school as experimental subjects. The basic status is shown in Table 1.

In the experiment, a video camera was used to record the detailed steps of the athletes in the long jump. The central axis of the transmission belt is marked with a square every 20 cm on the longitudinal axis of the belt. The size is 2.0 cm × 2.0 cm, and the shooting distance is 10.50 m. The width of the viewfinder can capture the athlete's entire body very well. The width is 1.50 m × 0.90 m, and the shutter speed is 1/250 s. The purpose of using a treadmill in shooting is to use the motion analysis used in calculating the horizontal support reaction force to obtain the specific speed during the take-off process of the long jump movement, which can be reflected by the treadmill, and the actual detection is the result of the horizontal speed and acceleration of the treadmill movement. A three-dimensional AT3 acceleration sensor is fixed on the athlete to replace the sword-like process with the torso and the sternum of the human body (including the limbs) and the specific situation of the vertical acceleration of the upper limbs during the head movement. The specific situation is shown in Figure 6.

### 3.2. An Experiment on the Relationship between the Muscle Torque Changes of the Hip, Knee, and Ankle Joints of the Take-Off Leg and the Leaping Speed

Until now, science and technology have not been able to directly and accurately measure the contraction force of human muscles and the specific contraction force. But through the corresponding measurement of dynamics, combined with the theory of computational mechanics, the torque caused by a muscle group in a joint movement can finally be obtained, that is, the degree of tension of the muscle torsion. The torque of the joint muscles indicates the degree of its strength muscle group. The active muscles (active muscles and antagonist muscles) that “control” the joint are the complete performance of all muscles in the entire joint. The role of muscle groups in sports and the nature of their activities have their own unique characteristics. When torque analysis is performed, successful and failed technical movements can be studied, or the skills of different athletes can be compared and analyzed, which can quantitatively reflect those functional status and functional characteristics of muscle groups that promote human movement.

The final long jump performance in the long jump is the distance from the center of the human body at the starting point, and to a large extent depends on the speed of ascent, that is, the speed of the athlete after the take-off action ends, which can lead to the final result of the long jump. The ascent speed is determined by the ability of the muscles, especially the strength and contraction of the joint muscles in the long jump. The size and torsion of the joint muscles can reflect its degree and nature. Therefore, it is necessary to discuss the ascent width and the width of the hip, knee, and ankle in depth. The relationship between jumping speed has been studied in depth. After many athletes and many tests, it was found that the maximum muscle duration and jumping speed of the hip, knee, and ankle muscles of the athlete's take-off leg are shown in Table 2.

After conducting related experiments, we respectively performed correlation analysis on the joint torque peak and the leaping speed to determine the degree of correlation between them. The specific results are shown in Table 3.

It can be seen from the above experimental results that the correlation coefficients between the maximum torque of the hip and ankle joints and the jumping speed are 0.514 and 0.523, respectively, which are significantly positively correlated with the peak point (*P* < 0.05). There is also a certain correlation between knee joint torque and leaping speed, there is a positive correlation (*r* = 0.439), but the correlation is not significant (*P* > 0.05).

In order to further study the relationship between joint muscle torque and jumping speed, the specific experiment is divided into two groups according to different jumping test speeds. The jumping speed of 8.32 m/s is the median of all test jumps, that is, 9 groups of experimental jumps (group A) with a take-off speed less than or equal to 8.32 m/s and the closing speed of the take-off speed of 10 test jumps. More than 8.32 m/s is assigned to another group (group B). Figures 7, 8, and 9 compare the muscle tension of the hip, knee, and ankle joints between the two groups and compare the maximum muscle values of the hip, knee, and ankle joints of the rising leg in two jumps.

### 3.3. The Characteristics of the Muscle Torque Changes of the Hip, Knee, and Ankle Joints in the Take-Off Leg

In order to further study the relationship between musculoskeletal momentum and jumping speed, based on the original experiment, the last jumping test was divided into two groups according to the jumping speed, and the *t*-test was aimed at the two groups of hip, knee, and ankle muscle torque samples and was used for the maximum value. The results in Table 4 show that the average peak duration of hip, knee, and ankle joints in group B is longer than that in group A, and the maximum length of hip and ankle muscles is significantly higher than the difference in group A (*P* < 0.05). It can be seen that the torque of the hip, knee, and ankle muscles is significantly correlated with the center of gravity of the ascent speed and is significantly positively correlated (*P* < 0.05). Observing the specific experimental conditions of the two groups, it can be seen that the higher the muscle torque, the higher the center of gravity speed, especially the hip and ankle muscle torque, which has a more significant impact on the flight speed and time in the long jump.

The pressure center of the foot is the point of action of the resultant force of the foot on the ground during the take-off process of the long jump movement, that is, the point of action of the three-dimensional support reaction force on the ground. Certain research and experimental data show that changes in the center of pressure will affect the effect of long jump to a certain extent. The greater the change in the pressure center, the worse the actual effect of the take-off action, and the worse the concentration of the athlete's effort, resulting in unsatisfactory final results. This experiment analyzes and discusses the relationship between the change of the plantar pressure displacement center and the lifting speed in multiple jump tests, and conducts in-depth research on the actual situation.

From Table 5, we can see the increase in the speed of the center of gravity for different jumps, and the overall trend of the change of the pressure center is decreasing. The change of the pressure center is between 51.26% and 74.35%. The center pressure of the foot in the two test jumps is shown in Figure 10.

## 4. Discussion

Based on the above experimental results, we found that the hip joint of the foot will produce greater hip joint stretching torque during the initial period of time and eccentric work, and joint expansion is very important during the entire exercise. The entire muscle group plays a vital role in the long jump. Within a period of time at the beginning of the take-off, the knee joint of the take-off center foot produces more flexion torque, indicating that the knee joint flexion group muscles contract, and the ability of the entire muscle group plays a role in the entire take-off movement, avoiding muscle damage to the back of the thigh. The degree of muscle tension and contraction of the hip, knee, and ankle joints of the take-off center leg is closely related to the human body weight. The greater the muscle torque, the higher the speed of lifting the center of gravity, especially the stretching torque of the hip and ankle joints has a great influence on the lifting speed, and it also has a very significant effect in the subsequent aerial exercise. The smaller the displacement of the pressure center, the higher the speed of the center of gravity, and the longer the subsequent flight time, which is very beneficial to the final good results. It can well improve the athlete's ability, increase the athlete's stability to support the upward trend, and ultimately have the effect of improving the jumping effect to achieve a longer distance.

## 5. Conclusions

In the initial stage of long jump take-off, the knee joint produces a large flexor torque, that is, the active contraction of the knee joint flexor muscle group, which is caused by the forward extension of the take-off foot and the impact of the large ground reaction force when landing. This feature should be given enough attention by coaches and athletes in training. Based on the multi-information fusion technology, this paper studies the special ability of the long jump take-off muscles, explores the working state of the relevant muscle groups in the long jump, and finds a suitable method to improve the take-off method for athletes and increase the athlete's vacancy. Time can ultimately achieve better results. Use multi-information fusion technology to conduct research, such as the information processing of the hip, knee, ankle muscle torque changes of the take-off leg, and analyze and process it under certain criteria to complete the required decision-making and estimation tasks. By comparing with the full run-up long jump, the results of the speed control test can better reflect the characteristics and laws of each joint muscle group of the take-off leg suitable for the special long jump. Ability test can become an effective means of long jump athletes' special ability test, assessment, and special strength training.

## Figures and Tables

**Figure 1:** The working principle of information fusion technology.

**Figure 2:** Multisource data fusion process.

**Figure 3:** Key technologies of multisource information fusion.

**Figure 4:** The four components of long jump.

**Figure 5:** Schematic diagram of human skeletal muscle hierarchy model.

**Figure 6:** Detailed schematic diagram of long jump take-off action.

**Figure 7:** Comparison diagram of hip joint muscle torque.

**Figure 8:** Schematic diagram of knee joint muscle torque comparison.

**Figure 9:** Schematic diagram of ankle joint torque comparison.

**Figure 10:** 001 and 012 test jump pressure center change curve.

**Table 1:** Basic situation of experimental subjects.

Numbering	Age	Height	Weight	Current grade	Best grade
1	21	1.74	69.5	6.51	6.81
2	22	1.82	73.5	7.16	7.46
3	23	1.75	55.4	7.34	7.50
4	22	1.74	65.5	7.04	7.40
5	22	1.70	65.0	6.57	6.95
6	21	1.72	65.4	6.55	6.98
7	22	1.73	68.0	6.59	7.02
8	21	1.76	69.0	6.82	7.12

**Table 2:** Take-off leg hip, knee, and ankle joint muscle torque changes and take-off speed.

Jump	Peak hip torque	Peak hip torque	Peak hip torque	Center of gravity rise speed
014	14.24	4.91	7.24	7.51
018	21.95	12.79	8.37	7.61
010	16.15	8.83	6.57	8.79
005	34.57	14.35	13.49	8.29
012	12.27	9.34	7.36	8.13
008	13.61	5.76	5.16	8.22
015	15.34	6.25	6.14	7.91

**Table 3:** Correlation analysis of take-off leg hip, knee, and ankle joint muscle torque peak and lift speed.

Statistics	Peak hip joint muscle moment and leaping speed	Knee joint muscle torque peak and leaping speed	Peak ankle muscle torque and lifting velocity
Correlation coefficient	0.514	0.439	0.523
*P*	0.062	0.134	0.021
*S*	0.576	0.573	0.544

**Table 4:** Comparison of peak muscle movements of the hip, knee and ankle joints in test jumps between groups A and B.

A			B		
Hip joint	Knee joint	Ankle joint	Hip joint	Knee joint	Ankle joint
14.24	4.59	7.56	22.04	10.16	11.58
21.95	12.61	7.89	35.21	18.59	9.29
16.15	8.26	7.16	27.65	9.16	16.53
37.45	14.35	15.24	19.87	6.29	6.49
12.75	5.49	5.48	23.15	28.16	10.27
32.16	9.46	10.26	29.24	11.54	15.39

**Table 5:** The results of the longitudinal displacement of the plantar pressure center and the rise speed.

Jump	Foot length	Longitudinal displacement of pressure center	Longitudinal displacement of pressure center as a percentage of foot length	Center of gravity rise speed
014	25.23	13.18	51.26	7.24
018	16.91	21.26	74.35	7.49
010	26.48	24.51	73.56	7.59
005	28.16	19.06	58.16	8.04
012	27.27	14.88	66.24	7.91
008	23.52	17.26	71.26	8.51
015	25.26	19.52	56.24	8.21

## Data Availability

No data were used to support this study.
